RETRACTED

# MicroRNA-153 Inhibits Osteosarcoma Cells Proliferation and Invasion by Targeting TGF-β2

**DOI:** 10.1371/journal.pone.0119225

**Published:** 2015-03-20

**Authors:** Guangfeng Niu, Bin Li, Li Sun, Chenggong An

**Affiliations:** 1 Department of Orthopaedics, Shandong Provincial Hospital affiliated to Shandong University, Shandong University, Jinan, P.R. China; 2 Department of Orthopaedics, Dingtao County Hospital, Dintao, P.R. China; Peking Union Medical College Hospital, CHINA

## Abstract

Increasing evidence indicates that microRNAs (miRNAs), a class of small noncoding RNAs, participate in almost every step of cellular processes. MiRNAs are aberrantly expressed in human cancers and contribute to cancer development and progression. Study of miRNAs may provide a new clue for understanding the mechanism of carcinogenesis and a new tool for cancer treatment. In the present study, miR-153 was downregulated in human osteosarcoma tissues and cell lines. Introduction of miR-153 mimics into the MG-63 cells inhibited cell proliferation and invasion. Our results further revealed that transforming growth factor beta 2 (TGF-β2) was negatively regulated by miR-153. Furthermore, overexpression of miR-153 decreased p-SMAD2, p-SMAD3, epidermal growth factor receptor (EGFR) and insulin-like growth factor binding protein-3 (IGFBP-3) expressions, which were the downstream signaling molecules of TGF-β. Furthermore, miRNA-153 suppressed TGF-β-mediated MG-63 proliferation and migration. Therefore, our results suggest that miR-153 may act as a tumor suppressor in osteosarcoma through targeting TGF-β2.

## Introduction

Osteosarcoma is the most common type of primary bone tumor in children and adolescents, accounting for approximately2.4% of all malignancies in pediatric patients[1–3]. Due to extensive advancements in diagnostic methods and therapeutic techniques, the 5-year survival rate of OS patients has largely improved over the past decades to about 60–70%[4–6]. Although many osteosarcoma patients initially respond to chemotherapy, patients with metastatic or recurrent disease has extremely poor survival outcomes[7,8]. Thus, it is urgent to identify the molecular mechanisms underlying osteosarcoma development and progression to optimize therapeutic options.

MicroRNAs (miRNAs) are a class of endogenous non-coding RNAs (about 22 nt), regulating gene expression by binding to the 3’untranslated region (UTR) of target mRNAs, thereby leading to their translational repression and/or degradation[9–12]. MiRNAs play a significant role in various biological processes, including cell proliferation, differentiation, migration, metabolism and apoptosis[13–15]. It has been well established that deregulated miRNAs play significant roles in cancer progression, including tumor development, growth, differentiation, invasion, metastasis, and angiogenesis[16–19]. Therefore, identification of specific miRNAs in cancers might provide potential therapeutic targets for cancer treatment.

RETRACTED

Previous studies have showed that miR-153 is involved in the progression of various cancers, including breast cancer, glioblastoma, ovarian, oral, colorectal, lung and prostate cancer[20–25]. The role or molecular mechanism of miR-153 in osteosarcoma is still unknown. In the present study, the expression of miR-153 was down regulated in osteosarcoma cells and tissues. The ectopic expression of miR-153 suppressed cell proliferation and invasion in osteosarcoma cells. Moreover, transforming growth factor (TGF)-β2 (TGF-β2) was confirmed as a new direct target of miR-153 in osteosarcoma, and miR-153 may suppress tumor growth and invasion by repressing the expression of TGF-β2. In conclusion, we supposed that miR-153 played significant role in osteosarcoma development and might be a promising therapeutic target for osteosarcoma.

## Materials and Methods

### Ethics Statement

All patients (patients’ parents on behalf of the children) agreed to participate in our study and gave written informed consent. Both this study and the consent were approved by the ethical board of the institute of The Shandong Provincial Hospital affiliated to Shandong University and complied with Declaration of the Helsinki.

### Tissues and cell lines

Twenty paired osteosarcoma and adjacent non-tumor tissues (located >3 cm from the tumor) were obtained from Shandong Provincial Hospital affiliated to Shandong University. All patients gave written informed consent. Both this study and the consent were approved by the ethics committee of our Hospital. Human osteosarcoma cell lines (HOS, Saos-2, MG-63, and U2OS), and the normal osteoblast cells (NHOst) were obtained from ATCC and cultured in Dulbecco’s modified Eagle’s medium (DMEM) at 37°Cwith5% CO2 (S1 Table).

### RNA extraction and quantitative real-time PCR

Total RNAs were extracted from the cells or tissues using the miRNA Isolation Kit (Ambion, TX, USA). Reverse transcriptions were performed using TakaraRNA PCR kit (Takara, China) in accordance with manufacturer’s instructions. To quantify the transcripts of genes, real-time PCR was performed by a SYBR Green Premix Ex Taq (Takara, Japan) on LightCycler 480 (Roche, Switzerland). U6 and GAPDH were the normalizing controls for miRNA and mRNA quantification, respectively (S2 Table).

### Western blot

Tissues or cells were lysed using ice-cold lysis buffer (50 mM Tris—HCl, pH7.0, 1%w/v SDS, 10%glycerol) and were centrifugated at 4°C. Subsequently, proteins in the supernatants were quantified. After being separated by10% SDS PAGE, the proteins were blotted onto nitrocellulose membrane (Amersham BioSciences, Buckinghamshire, UK). After being blocked with 10% nonfat milk in PBS for 1 hour, the membranes were immunoblotted with antibodies as indicated. Then the membranes were immunoblotted by HRP-linked secondary antibodies (Cell Signaling). The signals were detected by SuperSignal West Pico Chemiluminescent Substrate kit (Pierce, Rockford, IL, USA). Anti-p-SMAD2, SMAD2, p-SMAD3, SMAD3, EGFR, TGF-β2 and IGFBP-3, and glyceraldehydes 3-phosphate dehydrogenate (GAPDH) antibodies were obtained from Abcam Company (USA). Enhanced chemiluminescence (ECL, Amersham Pharmacia Biotech) system was used to visualize intensity of the bands, which were subsequently exposed.

RETRACTED

### Oligonucleotide and transfection

The miR-153mimics and scramble were synthesized by GenePharma (Shanghai, China) and transfected into cells until the final oligonucleotide concentration reached20 nmol/l. DharmaFECT1 reagent (Dharmacon, Austin, TX, USA) was used for all cell transfections.

### Cell proliferation and invasion assays

The viability of the cells was analyzed by CCK-8 (Dojindo; Kumamoto, Japan), conducted daily for 3 days. Viable cells were counted by absorbance measurements at 450 nm by auto microplate reader (infinite M200, Tecan, Austria). To determine tumor cell invasion, transwell chambers (8 μm pore size; Costar, Switzerland) were used. The transwells were prepared for an initial equilibrium by adding 0.6 ml of RPMI-1640 medium to the transwell chambers, in which the lower compartment was supplemented with 10% fetal bovine serum as a chemoattractant. The inserts were incubated with 1 mg/ml BD Matrigel Matrix (BD Biosciences, USA). Then the cells were suspended in 0.2 ml of fresh medium without fetal bovine serum, and added to the inserts. After being cultured for 24 h, cells on the upper surface of the membrane were removed by cotton buds. Cells on the lower surface of the inserts were stained with 0.1% crystal violet. The number of cells was counted under a light microscope. For each insert, 5 different random visual fields (× 200 magnification) were selected.

### Luciferase reporter assay

Luciferase reporter assay was done as described previously[26,27]. MG-63 cells were incubated at a density of 4000 cells per well in a 96-well plate and cultured for 24h. Subsequently, cells were transfected with 20 nM miR-153 mimics or scramble, 10 ng pGL3 and pGL3-TGF-β2–3’UTR or pGL3-TGF-β2–3’UTR Mut plasmid per well using Lipofectamine 2000, according to the manufacturer’s protocol. Using the Dual-Luciferase Reporter Assay (Promega), the relative luciferase activity was calculated after 48 h by normalizing Firefly luminescence to that of Renilla.

RETRACTED

### Statistical analysis

Data were presented as the mean ± standard deviation (SD) from three separate experiments. When comparing only two groups, Student’s t-test was used to calculate the differences. When comparing more than two groups, a one-way analysis of variance (ANOVA) was used. The differences between groups of metastasis in vivo were analyzed using the χ2 test. SPSS 16.0 (SPSS Inc., USA) was used to analyze all of the statistics. P<0.05 was considered as statistically significant.

## Result

### miR-153 was decreased in osteosarcoma tissues and cell lines

MiR-153 was decreased in osteosarcoma tissues compared with adjacentnon-tumor tissues (Fig. 1A and B). Moreover, the expression ofmiR-153 was decreased in four osteosarcoma cell lines (HOS, Saos-2, MG-63, and U2OS) compared with the normal osteoblast cells (NHOst) (Fig. 1C).

**Fig 1:** miR-153 was decreased in osteosarcoma tissues and cell line. (A) The miR-153 expression was determined by qRT-PCR in 20 paired osteosarcoma tissues and adjacent noncancerous tissues. The expression of miR-153 was normalized to U6 snRNA. Data is presented as log 2 of fold change of osteosarcoma tissues relative to non-tumor adjacent tissues. (B) Relative miR-153 expression levels in osteosarcoma tissues and their corresponding adjacent normal tissues. (C) The expression or miR-153 was analyzed in normal osteoblast cells (NHOst) and four OS cell lines (HOS, Saos-2, MG-63, and U2OS). ***p<0.001.

### Overexpression of miR-153 inhibited osteosarcoma cell proliferation and invasion

Increased expression of miR-153 was confirmed using qRT-PCR (Fig. 2A). Overexpression of miR-153decreased the proliferation of MG-63 cells (Fig. 2B). Furthermore, invasion analysis showed that miR-153 overexpression inhibited the invasive abilities of MG-63 cells (Fig. 2C).

**Fig 2:** Overexpression of miR-153 inhibited osteosarcoma cell proliferation and invasion. (A) qRT-PCR analysis of miR-153 expression after the transfection of miR-153 mimics or scramble or no treat. (B) The CCK8 assay used to evaluate the proliferation of the MG-63 cells after transferred with the miR-153 mimics or scramble or no treat. (C) Invasion analysis of the MG-63 cells after treatment with miRNA mimics, inhibitors or no treat; the relative ratio of invasive cells per field is shown on the right, ** p<0.01 and ***p<0.001.

### TGF-β2 was a direct target of miR-153 in osteosarcoma cells

TGF-β2 was predicted to be a target of miR-153 (Fig. 3A). The mRNA level of TGF-β2 was inhibited in the miR-153 mimic group (Fig. 3B). MiR-153 significantly suppressed the luciferase activity of WT 3’UTR, but not the MUT 3’UTR of TGF-β2 in MG-63 cells (Fig. 3C). Overexpression of miR-153 can also suppress TGF-β2 protein levels (Fig. 3D).

RETRACTED

**Fig 3:** TGF-β2 was a direct target of miR-153 in osteosarcoma cells. (A) Computer prediction of miR-153 binding sites in the 3’UTR of human TGF-β2 gene. (B) Expression of TGF-β2 mRNA was examined by qRT-PCR in MG-63 cells transfected with miR-153 mimic or the scramble mimics or no treat. The expression of TGF-β2 was normalized to GAPDH. (C) MG-63cells were co-transfected with miR-153 and WT or MUT 3’UTR of TGF-β2. (D) Protein level was detected by Western blotting in MG-63 cells transfected with miR-153 mimic or the scramble mimics or no treat. GAPDH was also detected as a loading control. ***p<0.001.

### MiR-153 overexpression repressed the p-SMAD2, p-SMAD3, EGFR and IGFBP-3 expression

p-SMAD2, p-SMAD3, EGFR and IGFBP-3 protein expression were downregulated with the treatment of miRNA-153 compared with scramble (Fig. 4A). TGF-β enhanced the mRNA and protein expression of IGFBP-3 and EGFR; meanwhile, following the miRNA-153 mimic treatment, EGFR and IGFBP-3 proteins and mRNAs were downregulated in the MG-63 cell line (Fig. 4B, C and D).

**Fig 4:** MiR-153 Overexpression repressed the p-SMAD2, p-SMAD3, EGFR and IGFBP-3 expression. The MG-63 was treated in serum-free medium in the presence and absence of TGF-β (50 ng/ml), scramble, or miRNA-153 mimic for 24 h. (A) Expression of p-SMAD2, t-SMAD2, p-SMAD3 and t-SMAD3 was detected using western blotting. GAPDH was used as a loading control. (B) Expression of EGFR and IGFBP-3 was detected using western blotting. GAPDH was used as a loading control. (C) The mRNA expression of EGFR was detected using qRT-PCR. The expression of MMP9 was normalized to GAPDH. (D) The mRNA Expression of IGFBP-3 was detected using qRT-PCR. The expression of EGFR was normalized to GAPDH.

### miR-153 is involved in TGF-β-induced osteosarcoma cell proliferation and invasion

TGF-β promoted the osteosarcoma cell proliferation and invasion. When miR-153 mimic and TGF-β was added into MG-63 cells, miR-153 mimic inhibited the TGF-β-induced osteosarcoma cell proliferation and invasion (Fig. 5A and B).

**Fig 5:** miR-153 is involved in TGF-β-induced osteosarcoma cell proliferation and invasion. The MG-63 was treated in serum-free medium in the presence and absence of TGF-β (50 ng/ml), scramble, or miRNA-153 mimic. (A) Invasion analysis of MG-63 cells treated with different combinations. The relative ratio of invasive cells per field is shown right. (B) Cell growth curves in MG-63 cells transfected with different combinations. ** p<0.01 and ***p<0.001.

RETRACTED

## Discussion

In the present study, the expression of miR-153 is down-regulated in osteosarcoma tissues and cell lines. Forced expression of miR-153 represses cell proliferation and invasion in MG-63 cells. Furthermore, TGF-β2 is identified as a direct target of miR-153. miR-153 overexpression can inhibit the expression of p-SMAD2, p-SMAD3, EGFR and IGFBP-3 expression, which are the downstream signaling molecules of TGF-β. Moreover, miR-153 is also involved in TGF-β-induced tumor proliferation and invasion. Therefore, our study, for the first time, identifies thatmiR-153 might be a tumor suppressor gene in the progression of osteosarcoma. However, further studies are still needed to investigate its roles in vivo.

Increasing studies have shown that miR-153 is involved in the progression of many cancers, including breast cancer, glioblastoma, ovarian, oral, colorectal, lung and prostate cancer[20–25]. Overexpression of miR-153 inhibited oral tumor cell metastasis via directly targeting SNAI1and ZEB2, acting as a tumor suppressor gene in glioblastoma stem cells[24]. Recently, Yuan et al. also found that miR-153 played a tumor suppressive role in lung cancer by suppressing AKT expression[22]. However, upregulation of miR-153 promoted colorectal cancer progression by increasing cell proliferation and down regulating PTEN [23,28]. These dual effects of miR-153 may be attributed to organ-specific actions and its different cellular contexts in tumors. To our knowledge, no information is available on the role or molecular mechanism of miR-153 in osteosarcoma. In our study, we investigated the expression of miR-153 in osteosarcoma clinical samples and identified that miR-153 was decreased in the osteosarcoma tissues. We also showed that miR-153 was down-regulated in the osteosarcoma cell lines in vitro. Furthermore, the functional role of miR-153 in osteosarcoma cell lines was investigated. Cell proliferation and invasion assays demonstrated that overexpression of miR-153 inhibited osteosarcoma cell proliferation and invasion. This was consistent with previous findings that overexpression of miR-153 suppressed glioblastoma (GBM) cell proliferation and GBM stem cell growth. These results suggest that miR-153 might act as a tumor suppressor gene whose down-regulation contributes to the progression and metastasis of osteosarcoma.

Recently, TGF-β, one of the most abundant growth factors stored and released by bone, has been proved to induce many cancer cells to proliferate[29–31]. TGF-β can promote cancer metastasis by regulating the composition of extracellular matrix, proteolysis and inflammatory responses[31–34]. Previous study showed that TGF-β stimulated MG-63 cell growth, introducing a novel regulatory role for IGFBP-3[35]. Previous study showed that TGF-β induced activation of the Raf/MAPK pathway[36]. Raf/MAPK pathway is closely associated with cell growth and cell invasion[37]. TGF-β2 also induced the IGFBP-3 expression, which can induce IGF action through high-affinity binding[30]. In osteosarcoma, TGF-β signaling is considered as a potential therapeutic target due to its involvement in epithelial mesenchymal transition and cell proliferation [38,39]. However, the underlying mechanisms are unclear. The ability of miR-153 to target TGF-β2in our data may provide one mechanism of post-transcriptional control of TGF-β2. This conclusion is supported by the following reasons: complementary sequence of miR-153 is identified in the 3’UTR of TGF-β2 mRNA; miR-153 overexpression led to a reduction at both mRNA and protein level of TGF-β2; reintroduction of miR-153inhibited 3’UTR luciferase report activity of TGF-β2and this effect was abolished by mutation of the miR-153 seed binding site. We further studied the functional roles of miRNA-153 in TGF-β signaling pathways. Our results showed that TGF-β could induce the p-SMAD2, p-SMAD3, EGFR and IGFBP-3 expression. Moreover, miRNA-153 overexpression repressed the p-SMAD2, p-SMAD3, EGFR and IGFBP-3 expression. These results indicate that miR-153 may function as a tumor suppressor partly by repressing TGF-β2 expression in osteosarcoma.

RETRACTED

Taken together, we demonstrated that miR-153 was downregulated in osteosarcoma cell lines and tissues. Overexpression of miR-153 resulted in inhibition of osteosarcoma cell proliferation and invasion. Further investigation revealed that TGF-β2 was a potential target of miR-153. Therefore, miR-153 may serve as a therapeutic target in osteosarcoma patients.

## Supporting Information

S1 Table Summary of clinicopathological parameters of patients with osteosarcoma. (DOCX)

S2 Table Primer sequence. (DOC)
